RETRACTED

# Qualitative Diagnosis of Liver Tumors Based on Ultrasound-Guided Automatic Biopsy

**DOI:** 10.1155/2021/8585887

**Published:** 2021-11-18

**Authors:** Bin Peng

**Affiliations:** The Central Hospital of Xiaogan, Xiaogan, Hubei 432000, China

## Abstract

The goal of this study was to see if automatic biopsy guided by ultrasound could be used to provide a qualitative diagnosis of a liver tumor. *Methods*. A total of 40 patients (101 focuses) were treated with automatic liver parenchyma biopsy under ultrasound guidance, and the correlation between pathological outcomes and ultrasound images was investigated. The lesion size in the observation group was compared to that in the control group using conventional ultrasound (*P* > 0.05), and there was no significant difference. Under contrast-enhanced ultrasound (CEUS), there was no statistically significant difference in lesion size between the observation and control groups (*P* > 0.05). The difference in lesion size between the conventional ultrasonography and CEUS observation groups was statistically significant (*P* 0.05). *Conclusion*. Ultrasound-guided automated biopsy of the liver parenchyma is a simple and effective procedure with fewer problems and a high diagnostic rate, and it deserves to be promoted clinically.

## 1. Introduction

In recent years, ultrasound-guided automated biopsy has become widely used in qualitative diagnosis of abdominal and pelvic space-occupying focus. The mortality rate of liver cancer has been rising in European and American countries in recent years. In China, the frequency of liver cancer remains high, and the overall incidence of liver cancer is expected to continue to climb. Hepatic hemangioma is a frequent benign liver tumor caused by a congenital blood vessel abnormality. Cavernous hemangioma, sclerosing hemangioma, hemangioendothelioma, and capillary hemangioma are the pathological classifications for hepatic hemangioma. The bulk of them are cavernous hemangiomas of the liver, and the last three are uncommon in clinic. Cavernous hemangioma is the most common type of hepatic hemangioma seen in clinic. Hemangioma is more frequent in the liver than in other organs. Because the tumors are so small, the majority of patients do not experience any symptoms. Liver cancer and liver hemangioma are two distinct diseases with distinct occurrences, progressions, treatments, and prognoses. As a result, in clinical work, determining the nature of focused focus detected in liver tests is quite useful in guiding treatment.

To date, surgical resection remains the most effective treatment for primary liver cancer. However, due to the influence of tumor scope, location, and liver function, the patients who can be given surgical treatment only account for about 20% of HCC patients, and the true success rate of surgical resection is only 30%, with a high recurrence rate after surgery [1]. It has been reported in the literature [2] that the sensitivity, specificity, and negative predictive value of benign and malignant tumors identified by morphology, site, boundary, and echo of the mass were 98%, 68%, and 99%, respectively. In addition, morphological changes of the mass after pressure from the probe can also help distinguish benign from malignant. Several diagnostic criteria have been proposed in the literature [3], including visualization, relative brightness, boundary uniformity, and lesion size of focus compared with elastic and two-dimensional images. These researchers found that the size of malignant tumors was larger than that of conventional ultrasound on elastic images. Literature [4] also proposed an elastic classification method based on the degree and distribution of strain, with the sensitivity, specificity, and accuracy of 87%, 90%, and 88%, respectively, for malignant diagnosis of breast tumor based on the elastic score of 3-4.

RETRACTED

Clinically, imaging examination methods such as ultrasonography and CT are used to diagnose liver space-occupying focus, although these approaches are not suitable for differentiating between benign and malignant foci [5]. Ultrasound-guided percutaneous needle biopsy has become a crucial diagnostic tool in clinical practice for qualitative diagnosis of liver space-occupying focus, thanks to the widespread use of interventional ultrasound in clinical practice. The manifestations of contrast-enhanced ultrasound (CEUS) of primary liver cancer are characteristic, mainly characterized by rapid overall enhancement of the arterial phase, which has a short duration and hypoechoic changes in the portal phase, showing the overall change of “fast in and fast out” [6]. However, the contrast manifestations of some primary liver cancers are atypical and difficult to distinguish from benign focus. On the basis of CEUS, we used the analysis software to analyze and compare the contrast-related data. To further explore the clinical application value of quantitative analysis of CEUS in qualitative diagnosis of liver tumors.

The current study is unique in that it is the first to use ultrasound-guided automatic biopsy for the qualitative diagnosis of abdominal and pelvic space-occupying foci. Its use in the qualitative diagnosis of liver tumors, on the other hand, is restricted. The goal of this research is to provide a reference for clinical qualitative diagnosis of liver tumors using ultrasound-guided automatic biopsy.

RETRACTED

## 2. Literature Review

### 2.1. Application Progress of Contrast-Enhanced Ultrasound in Interventional Ultrasound

In recent years, CEUS technology has become increasingly mature in the clinical diagnosis of many diseases. At the same time, interventional ultrasound has been widely used in clinical diagnosis. The close combination of CEUS and interventional ultrasound can find new advantages in clinical diagnosis.

#### 2.1.1. Application of Contrast-Enhanced Ultrasound in Percutaneous Transhepatic Biliary Puncture and Drainage

The most common causes for surgical jaundice in patients are biliary tract obstruction caused by inflammation, tumor, and calculus, which can cause increased pressure in small bile ducts and capillary bile ducts, dilation and rupture of lumens, and then bile overflow to small veins and reflux to increased blood circulation and biliary tract pressure. Patients gradually suffer from decreased hepatocyte function and increased heme, with clinical manifestations including obvious yellow staining of skin and sclera and skin pruritus.

Reasonable use of CEUS for accurate catheterization and drainage, judging the drainage range and predicting the drainage effect will have an important impact on the prognosis of patients. Some scholars used rabbit as the animal model for research and explored whether bile duct perfusion studied by CEUS via biliary tract is feasible. The rabbits were divided into four groups according to the concentration of diluted contrast agent. After administration, the perfusion of contrast agent in intrahepatic bile duct was observed, including whether the contrast agent 66 completely filled the bile duct, whether it overflowed and the satisfactory duration of imaging. Finally, it was concluded that it was feasible to apply CEUS to the biliary system to study bile duct perfusion, and it was considered that the concentration of contrast agent should not be too low, and the imaging effect was best with a concentration of 1/200 dilution [7].

#### 2.1.2. Application of Contrast-Enhanced Ultrasound in Percutaneous Nephrostomy

Congenital abnormalities of the urinary system, stones, tumors, trauma, and other common causes of urinary system obstruction, resulting in different degrees of kidney water, further development will cause renal damage, and even the late occurrence of uremia. In order to relieve the clinical symptoms of patients with hydronephrosis, control infection, improve renal function, or prepare for the removal of the cause of obstruction, percutaneous nephrostomy under the guidance of B ultrasound is often required to directly drain the urine to relieve the compression on the renal parenchyma [8].

RETRACTED

Percutaneous nephrostomy can not only protect the renal function but also greatly improve the quality of life of patients. Although percutaneous nephrostomy can be completed in most cases under the guidance of conventional ultrasound, the ability of conventional ultrasound is often limited when the puncture point and puncture direction are selected in some cases of mild hydronephrosis, upper calyx sputum production, and high kidney [9, 10]. Therefore, conventional ultrasound-guided percutaneous nephrostomy cannot fully meet the clinical needs, and it is necessary to explore a safer and more reliable puncture-catheter drainage method, so as to provide further help for finding the cause of obstruction.

#### 2.1.3. Application of Contrast-Enhanced Ultrasound in Radiofrequency Ablation of Liver Cancer

Tumor tissue ablation is another significant component of interventional ultrasound, and hepatocellular carcinoma ablation has been widely used in clinical practice. At present, the ablation treatment methods for liver cancer with more clinical applications include radio frequency activation (RFA), microwave coagulation activation (MWA), cryoablation and high intensity focused ultrasound activation (HIFU). The basic principle of most treatment methods is to destroy the tumor tissue using its unique physical characteristics to cause coagulation and necrosis of the tumor tissue for local treatment. Among them, RFA was carried out early and to a certain extent it was representative.

The efficacy of RFA in the treatment of liver cancer is also closely related to the tumor size. Therefore, we should decide whether RFA is feasible or not to improve the cure rate of RFA for liver cancer on the premise of fully understanding the lesion size. In the previous study [11], a total of 222 focuses were grouped and compared in 167 patients who met the treatment indications of RFA. Among the 81 cases with 110 focuses that underwent CEUS before RFA, and 86 cases with 112 focuses that did not undergo CUES before RFA, the results showed that seven new focuses were found during CEUS examination, which were not found in conventional ultrasound examination or enhanced CT examination. Moreover, 56.4% of the focuses were found to be larger than conventional ultrasound, and 49.1% of the focuses were more irregular in boundary than conventional examination.

Literature [12] A retrospective study was conducted to analyze 64 ablation cases. The subgroups in this study found that the residual tumor rate in the CEUS group at the end of treatment was 0%, while the residual tumor rate in the non-CEUS group was 16.7%. The results showed that performing CEUS immediately at the end of RFA treatment to evaluate the ablation effect could effectively reduce the incidence of residual tumors after thermal ablation, and provide accurate information for RFA operators to guide ablation treatment. Besides, a study evaluating the intraoperative application of CEUS found that CEUS can immediately evaluate the ablation effect, not only without increasing the patient's cost, but on the contrary, it can reduce the treatment cost for patients with liver cancer and alleviate the economic burden on patients [13].

RETRACTED

In summary, CEUS has broken the traditional concept that imaging of the target area can be achieved by injection of contrast agent through the external elbow vein, and imaging can also be provided with valuable information for clinical diagnosis and treatment by injection through non-vascular lacunar ducts. Ultrasound-guided therapy has been increasingly accepted and recognized clinically because of its advantages such as small trauma, no radiation, accuracy and real-time dynamics. Reasonable and standardized application of CEUS in interventional ultrasound diagnosis and treatment and playing the important role of interventional CEUS not only can improve the disease diagnosis efficiency, but also can efficiently guide clinical treatment, provide the most valuable information for clinical doctors and bring the least pain and maximum benefit to patients.

### 2.2. Pathogenesis of Liver Cancer

Primary liver cancer is one of the most common malignant tumors in China, coming in second only to lung cancer in terms of incidence. According to statistics, China has the highest incidence of liver cancer in the world, with more males than females. With recent advances in molecular biology, virology, and genetics, it is now widely assumed that primary liver cancer is caused by a combination of multifactor, multipathway, and multistep long-term effects, including external environmental carcinogenic factors as well as its own genetic factors.

#### 2.2.1. Virus Infection

There is a close relationship between hepatitis B virus (HBV) infection and the occurrence of hepatocellular carcinoma (HCC). The results of several epidemiological studies have shown that worldwide, with few exceptions, chronic HBV infection has great similarities with HCC occurrence regions [14, 15], and the incidence of HCC is also relatively low in regions with low HBV infection. The mechanism of direct carcinogenesis of HBV is that the integration of HBV genome into host cells causes the simultaneous destruction of HBV DNA sequence and host cell gene sequence, or the occurrence of reintegration, which leads to the activation of oncogenes and inactivation of tumor suppressor genes, leading to cell carcinogenesis. Chronic hepatitis B can cause liver fibrosis and uncontrolled hepatocyte growth, and monocytes present in inflammatory liver tissue can locally produce reactive oxygen species, which can promote the occurrence of liver cancer.

RETRACTED

Hepatitis C virus (HCV) has been proved by the research in China and abroad. Hepatitis C and B are the important causes of liver cancer. HBV is the main cause of liver cancer in developing countries, while HCV is the main cause in developed countries [16]. At present, it is generally believed that continuous infection is obtained due to HCV sequence variation and evasion of immune recognition and hepatocyte degeneration, necrosis, and regeneration occur repeatedly, leading to the accumulation of gene mutations. The C protein and NS3 structural region of HCV destroy the dynamic balance of cell proliferation by regulating the expression of related genes and participating in signal transduction regulation, leading to cell canceration [17].

#### 2.2.2. Aflatoxin

A large number of epidemiological investigations and laboratory studies have confirmed that the incidence of liver cancer has a graded correlation with the amount of aflatoxin intake, and HBV and aflatoxin have a synergistic carcinogenic effect [18]. At present, aflatoxin is considered to be closely related to the mutation of tumor suppressor gene p53. Researchers in China and abroad can detect p53 gene mutation in liver cancer patients with high aflatoxin exposure, and it mainly occurs at codons 249 and 254.

#### 2.2.3. Relationship between Alcohol, Tobacco, and Occurrence of Liver Cancer

Drinking alcohol mainly plays an auxiliary role in the occurrence of liver cancer. There is little evidence that alcohol itself is a carcinogen, but studies have shown a relationship between alcohol intake and the risk of liver cancer (OR): OR < 1 at low doses; The medium dose was OR > 1; Severe alcohol consumption increased the OR value by 2.75 times, and the OR value increased with the increase of drinking dose in a significant dose-response relationship [19].

The risk of liver cancer and liver cancer mortality caused by smoking increase with the increase of cigarette smoking, and there is a significant positive correlation between cigarette smoking and liver cancer [20]. There was a synergistic effect between alcohol consumption, smoking, and hepatitis B virus infection [21].

#### 2.2.4. Relationship between Genetic Factors and Occurrence of Liver Cancer

Epidemiological studies have shown that after exposure to the same environment, the genetic susceptibility of the exposed plays an important role in the pathogenesis of environmental factors. The genetic susceptibility indicators studied at present include

1. GST gene polymorphism, including GSTM1, GSTT1, GSTP1. Polymorphism in the coding sequence of GST gene may affect the carcinogenic function of the metabolic environment of the body [22].
2. Cytochrome P4501A gene polymorphism. It can cause a large amount of final carcinogen accumulation in the body, making the chance of final carcinogen binding to p53 gene greatly increased, resulting in p53 gene mutation [23].
3. Acetaldehyde dehydrogenase 2 gene polymorphism. It can affect alcohol metabolism, and the increased acetaldehyde concentration in the body can lead to an increased risk of hepatocellular carcinoma [24].

RETRACTED

#### 2.2.5. Relationship between *Helicobacter pylori* Infection and Hepatocellular Carcinoma

Studies outside China have found that *Helicobacter pylori* can cause chronic active hepatitis in some strains of mice and induce liver cancer in sensitive mice [25]. Making it the first time that bacterial infections have been linked to cancer. Of the 28 HCC specimens detected by PCR, 17 were positive for 16SrRNA gene of *Helicobacter pylori* (60.7%). Using the specific probe southern hybridization as a method for identifying *Helicobacter pylori*, the results showed that 60.7% of patients with primary liver cancer did experience infection with *Helicobacter pylori*, and sequencing results confirmed that the *Helicobacter pylori* 16SrRNA sequence in their liver cancer tissues shared 97.8% homology with *Helicobacter pylori*.

*Helicobacter pylori* reaches the liver through the portal vein, lymphatic circulation and other pathways, and is mostly distributed in the capillary bile duct between the hepatocytes, and the possible mechanism of cancer is:

1. *Helicobacter pylori* itself and its metabolites have hepatotoxic effect [26]
2. Inflammatory infections release cytokines that drive the cell cycle and increase the expression of endogenous associated antigens to cause abnormalities in cell proliferative kinetics

## 3. Experimental Part

### 3.1. Research Objects

The research subjects were primary and metastatic liver cancer patients who visited our hospital. All of them were clinically diagnosed (surgical pathology or biopsy pathology) and applied for ultrasound-guided radiofrequency ablation of liver tumors, a total of 40 cases with 101 focuses.

According to the consensus, inclusion and exclusion criteria for all cases were established and grouped according to the location of liver tumors and tumor volume, that is, research subjects were divided into two groups: treatment difficulties observation group (hereinafter referred to as the observation group) and control group, depending on whether liver tumors were difficult and complex to treat. There were 45 focuses in the observation group and 56 focuses in the control group.

  Inclusion criteria:
(1) Liver malignant tumors that cannot be resected by surgery or for which the patient voluntarily selects ultrasound-guided RFA treatment
(2) Patients with liver tumors had no vascular tumor thrombi or invasion of adjacent organs
(3) Liver function classification Child-Pugh Grade A or B
  Exclusion criteria
(1) Diffuse hepatocellular carcinoma
(2) Accompanied with vascular cancer thrombi or invasion of adjacent organs
(3) Child-pughc of liver function, which could not be improved after liver protection treatment
(4) Esophageal (gastric) variceal hemorrhage occurs within one month before treatment
(5) Irreversible coagulation disorder and severe hemogram abnormality with severe bleeding tendency
(6) Recalcitrant massive ascites, cachexia
(7) Active infection, especially inflammation of the biliary system
(8) Severe liver, kidney, heart, lung, brain, and other major organ failure
(9) Patients with disturbance of consciousness or inability to cooperate with therapy

RETRACTED

### 3.2. Experimental Installation

#### 3.2.1. Ultrasonic Instrument

The ultrasonic instrument used in this study was PHILIPS IU22. The device is a multifunctional color Doppler ultrasound diagnostic apparatus. Has the advantages of high image quality, powerful functions, simple operation, and the like. The PHILIPS iU22 has a fully digital xSTREAM host architecture that can handle multiple data streams simultaneously—real-time processing—and supports an ultrawideband beam transmitter. Fast operation, running more than 250 billion times per second, makes real-time processing possible in all modes, including real-time three-dimensional volumetric imaging.

#### 3.2.2. Contrast-Enhanced Ultrasound Agent

Sonovue, sulfur hexafluoride microbubbles for injection, manufactured by BRACCO, Italy, with a specification of 59 mg sulfur hexafluoride, was used. Before use, 5 mL normal saline for injection (0.9% NaCl) was injected with matching instruments, fully shaken and homogenized to obtain microbubble suspension for later use.

#### 3.2.3. Ultrasound-Guided Percutaneous Liver Puncture Biopsy Device

Italian PRE TruCut needle was used for biopsy, with a diameter of 20G, a length of 10 cm and a cutting groove length of 2 cm.

#### 3.2.4. Contrast-Enhanced Ultrasound Quantitative Analysis Software

QLAB CEUS Image Analysis Software is a new contrast analysis software released by PHILIPS, which can be run on personal computers and also used in various computer operating systems such as windows XP. Compared with the previous contrast analysis software, when using this software for CEUS, the acquisition of contrast images has the following requirements:

1. The settings of contrast conditions of ultrasonic instruments shall be adjusted according to the recommended use and adjustment requirements of different instruments, and the concentration of contrast agent in the circulating blood and the stability of microbubbles shall be maintained to the maximum extent, for example, the settings of two-dimensional gray scale gain, TGC, mechanical index (MI) and other parameters
2. For CEUS, the section image should be located on the largest section of the lesion and the image should be kept on the same section to the maximum extent
3. In order to minimize the images caused by breathing or probe jitter, the patient should be asked to maintain stable breathing as much as possible and keep the stability of the probe
4. The injection method of contrast agent should be bolus injection
5. Contrast images should be recorded continuously for at least 180 seconds

RETRACTED

### 3.3. Method

The technical route is shown in Figure 1:

#### 3.3.1. Conventional Ultrasonic Examination Method

A comprehensive scan of the liver was performed to confirm the focus's location and number, to fully comprehend the focus's size, morphology, internal echo structure, color blood flow signals, spectral characteristics, and the relationship between the focus and the surrounding important tissues and structures, as well as to measure and record the relevant data and store the static and dynamic imprints.

The description of routine ultrasound results of focal liver focus includes the following aspects:

*(1) The Size of the Lesion*. The maximum diameter was measured on that largest section shown in the lesion.

*(2) The Morphology of Focus*. The spherical or ellipsoidal shape of focal liver focus is defined as regular morphology, and it is called irregular morphology when the focus have no certain morphology and grow irregularly.

*(3) Echo Types of Focus*. The normal liver parenchyma echo was taken as the reference, and the normal spleen echo could be taken as the reference when the liver was accompanied with diffuse focus. A lesion with an echo similar to that of the lesion was defined as isoecho, and the lesion with an echo higher than that was defined as hyperecho, and that with an echo lower than that was defined as hypoecho.

*(4) The Boundary of the Lesion*. The focus with complete and continuous capsule and clear boundary with liver parenchyma were called with clear boundary, while the focus without obvious capsule or with discontinuous capsule and unclear boundary with liver parenchyma were called with unclear boundary.

*(5) Focal Blood Flow Signal*. There were two types according to the abundance of blood flow signals in and around the focus: linear and branched blood flow signals in and around the tumor focus were defined as the rich blood supply type, and no blood flow signal in the focus was defined as the less blood supply type.

*(6) Spectral Doppler Characteristic of Focus*. According to the RI, it was divided into two types, low resistance type (RI < 0.7) and high resistance type (RI > 0.7).

RETRACTED

#### 3.3.2. Contrast-Enhanced Ultrasound Targeted Spot Selection

The patient was in the supine or left lateral position, and the morphological characteristics of the lesion, including lesion size, echo, and boundary, were recorded using conventional two-dimensional ultrasound with an abdominal probe. Then color Doppler ultrasonography was performed to observe the blood supply. The contrast agent was prepared in advance. Using SonoVue produced by Bracco, Italy, 5 ml normal saline was injected into the SonoVue lyophilized powder bottle, and the bottle was vigorously shaken for several seconds until the lyophilized powder was completely and uniformly mixed to form an opalescent suspension.

Set the scan tool to contrast mode. A rapid bolus of 2.4 ml of SonoVue Suspension was injected through the superficial vein at the elbow and the tube was rinsed with 5 ml of normal saline. Timing was immediately started from the injection, and lesion enhancement characteristics in arterial phase, portal phase and delayed phase of the lesion were continuously observed in real time and dynamically according to the guidelines of the European Committee on Ultrasound Medicine and Biology for CEUS of the liver, and images were stored. According to the contrast results, the puncture biopsy was performed using the contrast-enhanced active region as the target.

#### 3.3.3. Ultrasound-Guided Percutaneous Liver Biopsy

Routine blood test and coagulation function examination before operation. The puncture biopsy can be performed only for patients who have no coagulation dysfunction or bleeding tendency and can tolerate the operation. Patients and their families were informed of the surgical risks and possible complications before surgery and informed consent was signed.

After routine disinfection and towel laying, the ultrasonic probe was covered with a sterile probe sleeve, a special puncture holder was mounted, and 2% lidocaine was used for local anesthesia. An 18G BARD needle biopsy was performed through the normal liver parenchyma to avoid large vessels. One to two needles were punctured conventionally. The average number of punctures was equal to the total number of punctures divided by the total number of punctures. The specimens obtained from the biopsy were fixed in 10% formaldehyde solution and then sent to the Pathology Department for histological examination. The ultrasound-guided puncture process is shown in Figure 2:

RETRACTED

#### 3.3.4. Contrast-Enhanced Ultrasound Analysis of Liver

The QLAB software will first be started and the contrast files stored on the CD will be imported into the analysis software. Secondly, various parameters of the software are set, and the settings of the parameters should be consistent with those of the ultrasound instrument during contrast. Selection of region of interest, which should include all the regions of the lesion as much as possible.

#### 3.3.5. Postoperative Observation and Treatment

After the patient's vital signs were stabilized, the stretcher was returned to the ward and he was told to stay in bed for 24 hours. Monitoring of blood pressure, oxygen saturation and other vital signs and abdominal conditions, focusing on observing whether there is a complication. Patients were routinely treated with related therapies such as hemostasis, analgesia, liver protection and anti-inflammation, and the changes of the disease conditions were monitored.

#### 3.3.6. Statistical Treatment

SPSS14.0 statistical software was used. Taking the pathological results as the gold standard, calculating the sensitivity, specificity, positive predictive value and negative predictive value of elastography in the diagnosis of liver malignant tumor; The Chi-square test was used to compare the accuracy of elastography in diagnosing malignant tumors ≤2 cm and >2 cm.

## 4. Result

### 4.1. Routine Ultrasound Observations

In the observation group, there were 45 focuses, with the largest lesion being 10.3 cm, and the smallest lesion being 0.7 cm, with the average size of (3.22 ± 2.51) cm. Among them, 33 focuses were located in special locations, including six adjacent to the diaphragm, 11 located under the liver capsule, four close to the gastrointestinal tract, three adjacent to the gallbladder, and 10 adjacent to the great vessels. In addition, there were 12 cases with the maximum diameter ≥5 cm. The composition of the difficult factors for focus in the observation group is shown in Figure 3.

In the control group, 56 focuses were identified, of which 4 focuses were newly detected by CEUS before RFA treatment and were not measured under conventional ultrasound before operation. Among the remaining 52 focuses, the largest lesion was 4.6 cm and the smallest was 0.3 cm, with an average of (23.35 ± 0.88) cm.

The average values of the lesion sizes in the observation group and the control group are compared, and the results are shown in Table 1. By rank sum test, *Z* = −0.714, and *P* = 0.476 > 0.05 indicated that there was no significant difference in the lesion sizes between the two groups when measured by conventional ultrasound.

RETRACTED

### 4.2. Test Results of Contrast-Enhanced Ultrasound

Preoperative CEUS evaluation was performed on 80 focuses. Satisfactory contrast images were obtained for 45 focuses in the observation group and 55 focuses in the control group, while repeated observation of one lesion in the control group could not obtain a satisfactory effect. Under contrast conditions, the average maximum diameter of 45 focuses in the observation group was (3.36 ± 2.27) cm, and that of 55 focuses in the control group was (2.43 ± 0.78) cm. The lesion sizes of the two groups were compared, and *Z* = −0.963, *P* = 0.357 > 0.05by rank sum test. There was no significant difference in lesion size between the two groups measured in the CEUS shape.

In the observation group, 53% (24/45) of the focuses were ≤3 cm, 18% (8/45) were between 3 cm and 5 cm, and the other 29% (9/45) were >5 cm.

In the control group, 84% (46/55) of the focuses were ≤3 cm, and 16% (9/55) of the focuses were within the range of 3 cm to 5 cm (Figure 4).

A total of 101 focuses were treated with RFA, and CEUS was performed immediately to observe the size of ablation focus. The average maximum diameter of 45 ablation focuses in the observation group was (3.98 ± 2.51) cm, and that of 56 ablation focuses in the control group was (3.22 ± 0.84) cm.

### 4.3. Comparison of Lesion Size Measurement Results Using Conventional Ultrasound and Contrast-Enhanced Ultrasound

The average size of 45 focuses in the observation group was (3.23 ± 2.45) cm under conventional ultrasound and (3.41 ± 2.23) cm under CEUS. *Z* = −2.801 and *P* = 0.003 < 0.05 in rank sum test, and there was statistical difference in the lesion sizes measured by the two methods. The lesion CEUS measurement in the observation group was larger than that under conventional ultrasound.

A total of 56 focuses were found in the control group. The paired analysis of conventional ultrasound and CEUS was performed on the 56 focuses in the control group. The average lesion size was (2.36 ± 0.88) cm under conventional ultrasound and (2.63 ± 0.87) cm under CEUS. *Z* = −4.177, *P* < 0.05 by rank sum test. There was statistical difference in the lesion sizes measured by the two methods. The lesion size measured by CEUS in the control group was larger than that measured by conventional ultrasound.

In the observation group, the CEUS measurement result of 64% (29/45) of all focuses was larger than the conventional ultrasound measurement result, 16% (7/45) of the focuses were consistent with the conventional ultrasound measurement result, and 20% (9/45) of the focuses were smaller than the conventional ultrasound measurement result (Figure 5).

RETRACTED

Among them, 68% (38/56) of the focuses in the control group had an increase in CEUS measurement of lesion diameter compared with the conventional ultrasound measurement, and 25% (14/56) of the focuses had the same measurement results under the two methods. Only 7% (4/56) of the focuses had CEUS measurement results smaller than the conventional ultrasound measurement (Figure 5).

### 4.4. Effect Evaluation

One month after RFA treatment of 101 focuses, CEUS follow-up was performed to evaluate the efficacy of biopsy. CEUS indicated that a total of 85 focuses were completely ablated, and the overall complete ablation rate was 85%.

Among the 45 focuses in the observation group, 33 focuses were completely ablated, and 12 focuses were not completely ablated, with the complete ablation rate of 73.3%. In the control group, 48 of the 56 focuses were completely ablated, and eight focuses were not completely ablated. The complete ablation rate was 85.7% (Figure 6).

The complete ablation rate of focus between the two groups was compared. Although the complete ablation rate in the observation group was slightly lower than that in the control group, according to the chi-square test, *χ*^2^ = 0.407, and *P* = 0.516 > 0.05 indicated that there was no significant difference in the complete ablation rate between the two groups.

### 4.5. Patient Serum AFP Content Results

The patients with primary liver cancer were followed up for serum AFP content one month after operation and compared with those before operation. The results are shown in Figure 7.

Among the 13 cases of primary liver cancer in the observation group, AFP was always in the normal range in two patients, declined to varying degrees in eight patients, increased in four patients, and the level of AFP in one patient was the same as that before surgery.

In the control group, including 22 patients with primary liver cancer, the serum AFP values of six patients were consistent within the normal range, 10 patients experienced different degrees of AFP decline, five patients had higher AFP than before, and one patient was the same as the preoperative AFP.

### 4.6. Follow-Up of Survival Rate and Local Recurrence Rate after Surgical Treatment

The follow-up results of survival rate and local recurrence rate after treatment are shown in Figure 8.

This study was started in October 2019, and the complete case follow-up was conducted until January 2020. The survival rate and local recurrence rate of 101 patients with liver cancer treated by ultrasound-guided automatic biopsy were followed up for half a year and one year.

RETRACTED

In the observation group, the half-year and one-year survival rates of 45 patients were 78% (35/45) and 69% (31/45), respectively, and the local recurrence rates were 11% (5/45) and 18% (8/45), respectively.

In the control group, the half-year and one-year survival rates of 56 patients were 80% (46/56) and 75% (42/56), respectively, and the local recurrence rates were 7% (4/56) and 11% (6/56), respectively.

## 5. Discussion

During CEUS of the normal liver, the microbubble contrast agent was injected through the peripheral vein and entered the abdominal aorta through the pulmonary circulation, and a part of the microbubbles traveled from the abdominal aorta to the hepatic artery, where their introduction led to enhanced blood flow in the hepatic arterial system (early enhancement). Some microvesicles: transabdominal artery-splenic artery-splenic vein-portal vein; Through superior mesenteric artery-superior mesenteric vein-portal vein, liver entry results in increased flow (delayed enhancement) in the portal system. Primary liver cancer is a multi-vascular malignant tumor, and 90% of its blood supply is derived from the hepatic artery. Moreover, tumor cells can secrete angiogenic factors, stimulate neoangiogenesis, and have abnormal anastomosis with arterioles and venules. Deformation, shift, abnormal proliferation, vascular encircling, arteriovenous fistula, etc. of the tissue and vessels can be seen from the tissue morphology. The peripheral liver parenchyma was mainly supplied by portal vein.

A large number of studies have shown that angiogenesis is the prerequisite and basis for tumor growth and metastasis. Malignant tumors without neovascularization are usually in a semi-dormant state, limited to the primary site, and grow slowly. In the pre-vascular stage where solid tumors are formed, the primary tumors are usually 1–3 mm in diameter and the number of cells is limited to 106. The focus is in a static state for a long time, such as carcinoma in situ. Once the angiogenesis enters the late vascular stage, the tumor will grow uncontrollably, and the tumor volume can reach 10,000-20,000 times of the original size within two weeks, while a large number of tumor cells metastasize to the distant via blood vessels [27].

Transhepatic biopsy can not only identify the benign and malignant focus, but also carry out pathological classification, understand the cell morphology, tissue structure characteristics and differentiation degree, identify the malignant tumor as primary or metastatic, and guide clinical analysis of the etiology and treatment of various benign focus. Another study [28] has revealed that the size, location of liver cancer focus and the background of liver cirrhosis are the main causes of missed diagnosis by conventional ultrasound. Based on the above existing problems, it is not enough to rely on conventional ultrasound to evaluate the basic situation of the focus in liver malignant tumors before RFA treatment. It is necessary to further understand the true size, boundary range, location and adjacent relationship as well as the blood supply characteristics of the focus through other methods.

RETRACTED

The tissues obtained from ultrasound-guided needle biopsy are only a small part of the diseased tissues, which cannot completely represent the whole lesion. The puncture pathological results of different regions within the same lesion may be completely different. Therefore, detecting positive and representative diseased tissues by needle biopsy is the key to improving the success rate of needle biopsy, the positive rate of needle biopsy, the diagnostic coincidence rate of needle biopsy and the diagnostic accuracy of malignant focus. CEUS increases the blood supply information of liver space-occupying focus and helps to judge whether the focus are active or not. The blood supply of some hepatic space-occupying focus is not rich, and conventional ultrasound cannot meet the needs of the diagnosis of the focus and the evaluation of curative effects after treatment. The active tissue can be determined as soon as the contrast-enhanced area on CEUS is present, while the less active part shows mild enhancement in the arterial phase, and the non-active part shows no enhancement. CEUS can sensitively and delicately provide the internal microvascular distribution of liver space-occupying focus and judge the carcinomatous residue and recurrence of liver cancer after treatment, which is clinically of great significance.

Tumor angiogenesis plays an important role in the pathogenesis of tumors. Malignant tumors can secrete tumor angiogenic factors, and under their stimulation, tumors and surrounding tissues begin to produce new blood vessels, which are different from those of benign tumors in morphology, quantity and function. Some studies have applied the information technology [29] to observe the morphology of new blood vessels of hepatocellular carcinoma tumors, and the results show that the distribution of new blood vessels is disordered. The above pathological characteristics of tumor blood vessels led to abnormal tumor blood perfusion, and CEUS as a blood pool tracer imaging provided the theoretical basis for reflecting the true size of the lesion.

In this clinical study, the rank sum test was used to compare the lesion sizes of the two groups under conventional ultrasound and CEUS, and *P* > 0.05 meant that there was no significant difference in the lesion sizes between the two groups. However, in the treatment observation group, the largest diameter of tumors in seven of the 45 focuses was >cm, while all focuses in the control group were <5 cm. For analysis, there was no statistical difference in lesion size between the two groups probably due to the small sample size. If the sample size of focus with the largest diameter >5 cm was increased, the focus in the observation group would likely be larger than those in the control group.

RETRACTED

In this study, three cases of liver cancer CEUS showed atypical manifestations, and no significant contrast agent regression was observed in the portal venous phase and the delayed phase. The puncture pathological results of these cases confirmed highly differentiated liver cancer, while 25 cases of CEUS showed typical “fast-forward and fast-out” liver cancer. The puncture pathological results confirmed medium-to low-differentiated liver cancer. These differences reflect the sequential changes in hemodynamics during the formation of HCC, namely, with the increase of the malignancy of the nodules, the portal blood supply will gradually decrease and the arterial blood supply will gradually increase. In addition, CEUS parameter values of benign and malignant focus overlapped in some parts of the study, and it is difficult to identify the nature of the lesion in this case by only relying on the parameter values. These cases deserve further study in the future.

## 6. Conclusion

For qualitative diagnosis of liver tumors, ultrasound-guided automatic biopsy is an effective method with fewer complications and a high diagnosis rate. This technique is deserving of further clinical promotion due to its ease of use, high sampling quality, and lack of pain for patients. Furthermore, for nodular foci in the liver that are difficult to characterize with routine imaging and laboratory examination, clinicians should consider ultrasound-guided automatic biopsy as the first alternative qualitative diagnosis method.

## Figures and Tables

**Figure 1:** Method road map.

**Figure 2:** Ultrasound-guided puncture process.

**Figure 3:** Schematic diagram of constitution of lesion difficult factors in observation group.

**Figure 4:** Schematic diagram of lesion size distribution in two groups of CEUS.

**Figure 5:** Comparison between CEUS measurement and conventional ultrasound measurement in two groups.

**Figure 6:** Schematic diagram of ablation efficacy evaluated by CEUS in two groups one month after treatment.

**Figure 7:** Results of serum AFP content in patients with primary liver cancer after one month follow-up.

RETRACTED

**Figure 8:** Follow-up of survival rate and local recurrence rate after treatment.

**Table 1:** Under conventional ultrasound, the average value of the maximum diameter of the observation group was compared with that of the control group.

	Observation group (*n* = 45)	Control group (*n* = 56).	*Z*	*P*
Measurement under conventional ultrasound.	3.24 ± 2.17	2.36 ± 0.87	−0.714	0.476

## Data Availability

The data used to support the findings of this study are included within the article.
